# Target Recognition of SAR Images Based on SVM and KSRC

**DOI:** 10.1155/2021/4322678

**Published:** 2021-10-31

**Authors:** Haiyan Zhao

**Affiliations:** School of Information Science and Engineering, Tianjin Tianshi College, Tianjin 301700, China

## Abstract

A synthetic aperture radar (SAR) target recognition method combining linear and nonlinear feature extraction and classifiers is proposed. The principal component analysis (PCA) and kernel PCA (KPCA) are used to extract feature vectors of the original SAR image, respectively, which are classical and reliable feature extraction algorithms. In addition, KPCA can effectively make up for the weak linear description ability of PCA. Afterwards, support vector machine (SVM) and kernel sparse representation-based classification (KSRC) are used to classify the KPCA and PCA feature vectors, respectively. Similar to the idea of feature extraction, KSRC mainly introduces kernel functions to improve the processing and classification capabilities of nonlinear data. Through the combination of linear and nonlinear features and classifiers, the internal data structure of SAR images and the correspondence between test and training samples can be better investigated. In the experiment, the performance of the proposed method is tested based on the MSTAR dataset. The results show the effectiveness and robustness of the proposed method.

## 1. Introduction

Synthetic aperture radar (SAR) can realize all-day and all-weather reconnaissance through high-resolution remote imaging. The intelligent interpretation of massive SAR images has become a research focus. SAR target recognition aims to confirm the category of the target of interest in the SAR image, mainly by combining feature extraction and classifier [1]. Feature extraction is employed to achieve dimensionality reduction and compression of high-dimensional SAR images, thereby improving the efficiency and accuracy of subsequent classification. Physically relevant features including target region, boundary, and shadow could provide intuitive descriptions for the targets [2–6]. Data analysis algorithms represented by principal component analysis (PCA) and linear discriminant analysis (LDA) [7, 8] have been widely used in SAR image feature extraction and target recognition. And their effectiveness has been verified by experiments. Later, with the popularity of manifold learning algorithms [9–11], new feature extraction methods such as nonnegative matrix factorization (NMF) [9] further improved the target classification performance. However, these methods are basically based on linear decompositions, and it is not sufficient to investigate the inherent complex manifold structure of SAR images. As a remedy, researchers have improved the nonlinear processing performance of these linear feature extraction methods by introducing kernel functions. A typical representative is kernel PCA (KPCA) [8]. Many signal decomposition algorithms including wavelet analysis, monogenic signal, and empirical mode decomposition have also been successfully applied to SAR target recognition [12–15]. Besides, the scattering center features were popular in the design of SAR target recognition methods [16–18]. The classifiers design appropriate classification strategies for the extracted features to output the target label of the test sample. At present, a rich set of classifiers are available in SAR target recognition, including the K nearest neighbor (KNN) classifier [7], support vector machine (SVM) [19–21], and sparse representation-based classification (SRC) [22–27]. Recently, many SAR target recognition methods were developed based on the deep learning tools, among which the convolutional neural network (CNN) is a typical representative [28–35]. The design of the classifier also needs to consider the nonlinear characteristics of feature extraction. Specifically, when the extracted features do not have nonlinearity, it is necessary to improve the overall nonlinear processing ability of the recognition algorithm by adding nonlinear characteristics to the classifier. On the contrary, when the extracted features take into account the nonlinearity of the SAR image, the classifier part can weaken the demand for the nonlinearity. In this way, the advantages of extracted feature and employed classifier can be combined to enhance the classification performance.

Based on the above analysis, this paper proposes a SAR target recognition method that combines linear and nonlinear feature extraction and classification. First, PCA and KPCA are used to investigate the linear and nonlinear characteristics of the original SAR image to achieve a comprehensive description of the pixel distribution. PCA is a classic feature dimensionality reduction algorithm, which has good adaptability and robustness. The disadvantage is that PCA has relatively low processing capabilities for nonlinear data. KPCA improves the nonlinear ability of classic PCA by introducing the kernel function, so it is complementary to PCA. In the classification stage, SVM and Kernel SRC (KSRC) [36] are used to classify KPCA and PCA feature vectors, respectively. KSRC is an extension of SRC in the kernel space, which enhances the nonlinear ability of the classification algorithm by designing a suitable kernel function. Finally, the similarity vectors output by the two are reliably fused by linear weighting [37–40], and the target category is determined according to the fused result. This paper effectively combines the advantages of linear and nonlinear features and classifiers to improve the robustness of the SAR target recognition method. In order to test the proposed method, experiments are carried out based on the MSTAR dataset. The experimental results show the effectiveness of the proposed method.

## 2. Feature Extraction

As an important data analysis algorithm in pattern recognition, PCA has been widely used in SAR image feature extraction [7, 8]. The basic idea is to obtain a set of projection bases to maintain the maximum amount of information while removing redundant information. As a supervised feature extraction method, PCA needs the support of rich training samples. **X**={**x**_1_, **x**_2_,…, **x**_**n**_} is recorded as the training sample set, where **x**_**i**_ ∈ R^*d*^,  *i*=1,2,…, *n*, and the mean vector of the training samples is calculated as follows:

(1) $$\begin{array}{c} \bar{x}=\frac{1}{n}\sum_{i=1}^{n}x_{i}. \end{array}$$

Then, the covariance matrix of **X** is obtained as follows:

(2) $$\begin{array}{c} Q=\sum_{i=1}^{n}{\left(x_{i}-\bar{x}\right)}^{T}\left(x_{i}-\bar{x}\right). \end{array}$$

The eigenvalue decomposition is performed on **Q** as follows:

(3) $$\begin{array}{c} \left[V,D\right]=\text{eig}\left(Q\right). \end{array}$$

In equation (3), the eigenvalues and eigenvectors of **Q** are stored in the vector **V** and matrix **D**, respectively. The eigenvalues in **V** are arranged from large to small, and several eigenvectors corresponding to the largest eigenvalues are selected to construct the projection matrix of PCA.

KPCA is the expansion of PCA in the kernel space. By introducing an appropriate kernel function in the vector inner product calculation process, the nonlinear ability of the feature extraction method can be effectively improved [8]. Commonly used kernel functions include Gaussian kernel function, polynomial kernel function, and logarithmic kernel function.

## 3. Classifiers

### 3.1. SVM

SVM was first developed for two-class classification problem. By minimizing the defined structural risk, a hyperplane can be optimized to separate two types of patterns. Afterwards, for an input sample *x*, the decision by SVM is made as follows:

(4) $$\begin{array}{c} w^{T}\cdot \phi \left(x\right)+b=0, \end{array}$$

where *w* is vector containing the weight coefficients of SVM, which are related to the properties of the hyperplane; *ϕ*(*·*) is the kernel function for different kinds of nonlinear cases; and *b* is the bias.

With the demand for multiclass classification tasks, the traditional SVM was extended to process multiple types of patterns using strategies like “one-to-one” and “one-to-many.” Specifically, some mature toolboxes, e.g., LIBSVM [41], were developed to flexibly use SVM for different kinds of problems including pattern recognition and regression. In the field of SAR target recognition, SVM was widely used and the performance was validated. However, it also should be noted that the nonlinear processing capability of SVM is limited, and the robustness to nuisance situations like noises and occlusions is not good enough.

### 3.2. KSRC

SRC was developed based on compressive sensing theory and applied linear representation to data processing. At first, a global dictionary, i.e., *A*=[*A*^1^, *A*^2^,…, *A*^*C*^] ∈ *R*^*d*×*N*^, is established, where *A*^*i*^ ∈ *R*^*d*×*N*_*i*_^,  *i*=1,2,…, *C* includes the training samples from the *i*th class. Then, for the test sample *y*, the sparse representation is described as follows:

(5) $$\begin{array}{c} \hat{\alpha }=\arg\min{\left\|\alpha \right\|}_{0}\text{s.t.}{\left\|y-A\alpha \right\|}_{2}^{2}\leq \varepsilon , \end{array}$$

where *α* contains the coefficients to be solved and *ε* is the threshold for reconstruction error.

The *ℓ*_0_ norm in equation (5) makes the optimization tasks a nonconvex one, which is difficult to be solved. As a remedy, the *ℓ*_1_ norm was employed to replace *ℓ*_0_ norm as an approximation so the problem can be solved smoothly. In addition, other algorithms like orthogonal matching pursuit algorithm (OMP) and Bayesian compressive sensing (BCS) can also be employed to handle the problem to find the approaching solutions. With the estimated sparse coefficients, the decision by SRC is made as follows:

(6) $$\begin{array}{c} r\left(i\right)={\left\|y-A_{i}{\hat{\alpha }}_{i}\right\|}_{2}^{2},\;i=1,2,\ldots ,C,\\ \text{identity}\left(y\right)=\underset{i}{\arg\min}\left(r\left(i\right)\right), \end{array}$$

where ${\hat{\alpha }}_{i}$ denotes the coefficients related to the *i*th training class, which are extracted from $\hat{\alpha }$; *r*(*i*),  *i*=1,2,…, *C* is the calculated reconstruction error.

Similar to the idea of KPCA, KSRC introduces the corresponding kernel function in the sparse representation process, thereby improving the nonlinear processing ability of the classifier. The specific process can be found in literature [36]. By using KSRC, the nonlinear processing capability in the classification stage can be improved. Therefore, it can cooperate with the extracted features to enhance the final classification performance.

### 3.3. Target Recognition

In order to fully combine the advantages of linear and nonlinear features and classifiers, this paper adopts the idea of weighted fusion to make the final decision. For the reconstruction error results output by KSRC, this paper first transforms them with the following equation:

(7) $$\begin{array}{c} s\left(i\right)=\frac{1/\left(i\right)}{\sum_{j=1}^{C}1/r\left(i\right)},\;i=1,2,\ldots ,C, \end{array}$$

where *r*(*i*), *i*=1,2,…, *C* represents the reconstruction error of each category and *s*(*i*) represents the similarity between the test sample and each category. The smaller the reconstruction error of a certain category, the higher the similarity between the test sample and its category. At this time, the output result of KSRC has the same properties as SVM and can be used for subsequent weighted fusion.

Denoting the similarity vectors corresponding to SVM and KSRC as *s*_1_(*i*) and *s*_2_(*i*), respectively, the final similarity is obtained by linear weighting fusion as follows:

(8) $$\begin{array}{c} fs\left(i\right)=w_{1}s_{1}\left(i\right)+w_{2}s_{2}\left(i\right). \end{array}$$

In equation (8), *w*_1_ and *w*_2_ represent the weight and *fs*(*i*) is the similarity after fusion. Under the condition of very limited prior information, this paper sets *w*_1_=*w*_2_=0.5, assuming that both have the same importance.

Based on the above analysis, the basic process of the SAR target recognition method proposed in this paper can be summarized into the following steps.

Step 1. PCA and KPCA are used to extract features of all training samples and test samples
Step 2. SVM is used to classify KPCA feature vector and KSRC is used to classify PCA feature vector
Step 3. Based on linear weighted fusion, the similarities from SVM and KSRC output are fused
Step 4. The target label of the test sample is determined according to the fusion similarity result

## 4. Experiments and Analysis

### 4.1. MSTAR Dataset

The MSTAR dataset is currently the most authoritative dataset for validating SAR target recognition methods. It collects SAR images of ten types of ground vehicle targets, which provides effective data resources for multiclass recognition tasks. Both the optical and SAR images of the targets are observed in Figure 1. The MSTAR dataset can provide a variety of experimental settings for comprehensive testing of SAR target recognition methods including the standard operating condition (SOC) and extended operating conditions (EOC). In order to quantitatively evaluate the proposed method, several types of comparison methods are set up in the experiment, as follows. Comparison Method 1 uses SVM as the classifier and PCA for feature extraction. Comparison Method 2 uses SRC as the classifier and KPCA for feature extraction. Comparison Method 3 uses KSRC as the classifier and PCA for feature extraction. It can be seen that the Comparison Method 1 and the Comparison Method 3 are part of the developed method in this paper.

### 4.2. Results and Analysis

#### 4.2.1. SOC

SOC is first considered as a basic situation with the experimental setup shown in Table 1. Ten targets are involved, among which the training and test samples of BMP2 and T72 have some configuration variances.  Figure 2 shows the confusion matrix of the proposed method on ten types of targets. Among them, the horizontal and vertical coordinates correspond to the actual target category and the target category predicted by the proposed method, respectively. Therefore, the elements on the diagonal are the correct recognition rates of various targets. It can be seen that all ten types of targets can be correctly classified with a probability of more than 98%, and the final average recognition rate reaches 99.02%. The comparison of the average recognition rate of various methods to ten types of targets is shown in Table 2. The method in this paper is better than the three types of comparison methods, which proves its effectiveness. Compared with Comparison Method 2 and Comparison Method 3, the method in this paper effectively improves the final recognition performance through the linear weighting method on their fusion results and verifies the advantages of the proposed method in combining linear and nonlinear features.

#### 4.2.2. Configuration Variance

The same type of target may include different configurations (such as BMP2 and T72 in Table 1). In addition, as can be seen from the confusion matrix in Figure 1, the configuration variance also leads to a relatively low recognition rate for BMP2 and T72 targets. Therefore, it is a challenging problem to handle the configuration variance in SAR target recognition. This experiment uses the training and test sets shown in Table 3, in which the training and test sets of the BMP2 and T72 targets have completely different configurations. The average recognition rates of various methods under the condition of configuration variance are shown in Table 4. The method in this paper has achieved an average recognition rate of 96.24%, which is higher than those of the other methods. The results verify its strongest robustness to configuration variance. In this situation, the configuration differences between the training and test samples can be approached in the nonlinear space. By combining the linear and nonlinear features and classifiers, the overall robustness to configuration variance can be improved.

#### 4.2.3. Depression Angle Variance

The change of the depression angle will cause the SAR image of the same target to appear with more significant difference. In order to test the performance of the proposed method under the condition of changing depression angles, this experiment sets up the training and test sets shown in Table 5. Among them, the training set is 2S1, BDRM2, and ZSU23/4 three types of SAR images at an elevation angle of 17°, and the test set is from an elevation angle of 30° and 45°, respectively. The average recognition rates of different methods at two depression angles are shown and compared in Table 6. It can be seen that the method in this paper is significantly better than the comparison method at the two depression angles, fully verifying its robustness to depression angle variance. Under depression angle variance, there are some nonlinear changes or divergences between the training and test samples. The proposed method fully considers the possible nonlinear characteristics during feature extraction and classification so the capability to handle depression angle variance can be improved.

#### 4.2.4. Noise Corruption

SAR images measured in real environments are often affected by noise, resulting in low signal-to-noise ratio (SNR). At this time, the problem of SAR target recognition under noise interference is more challenging. On the basis of the original MSTAR dataset, this paper simulates the generation of noise samples according to the ideas in [17, 42]. The basic process is described as follows. First, the noise energy is decided based on the pixel energy of the original SAR image and the SNR of the expected noisy sample. Then, the noise data are generated based on the form of additive white Gaussian noise. Finally, the noise data are added to the original image, so the noisy image corresponding to the preset SNR is obtained. For the constructed noise test sample set, this paper conducts tests on various methods and obtains the results shown in Figure 3. It can be seen that the noise level has a great influence on the recognition performance of various methods. In comparison, the downward trend of the proposed method's recognition rate curve is the slowest, showing its stronger noise robustness.

## 5. Conclusion

This paper designs a SAR target recognition method by combining linear and nonlinear features and classifiers. PCA and KPCA are used to extract the linear and nonlinear features of the original SAR image. SVM and KSRC are used to classify the features extracted by KPCA and PCA, respectively. Finally, the linear weighting strategy is used to effectively fuse the results of SVM and KSRC to improve the robustness of decision-making. Based on the MSTAR dataset, experiments are carried out under four typical conditions of SOC, configuration variance, depression angle variance, and noise corruption. The results show the effectiveness of the proposed method.

## Figures and Tables

**Figure 1:** Images of targets to be classified: (a) BMP2; (b) BTR70; (c) T72; (d) T62; (e) BRDM2; (f) BTR60; (g) ZSU23/4; (h) D7; (i) ZIL131; (j) 2S1.

**Figure 2:** Confusion matrix achieved by the proposed method [22].

**Figure 3:** Performance of different methods under noise corruption.

**Table 1:** Training and test samples under SOC [6].

Class	Training set	Test set
BMP2	233 (Sn_9563)	195 (Sn_9563) 196 (Sn_9566) 196 (Sn_c21)
BTR70	233 (Sn_c71)	196 (Sn_c71)
T72	232 (Sn_132)	196 (Sn_132) 195 (Sn_812) 191 (Sn_s7)
T62	299	273
BRDM2	298	274
BTR60	256	195
ZSU23/4	299	274
D7	299	274
ZIL131	299	274
2S1	299	274

**Table 2:** Average recognition rates under SOC.

Method type	Average recognition rate (%)
Proposed	99.02
Comparison Method 1	97.12
Comparison Method 2	97.53
Comparison Method 3	97.64

**Table 3:** Training and test samples under different configurations.

Class	Training set	Test set
BMP2	233 (Sn_9563)	196 (Sn_9566) 196 (Sn_c21)
BTR70	233 (Sn_c71)	196 (Sn_c71)
T72	232 (Sn_132)	195 (Sn_812) 191 (Sn_s7)

**Table 4:** Classification results under configuration differences.

Method type	Average recognition rate (%)
Proposed	97.64
Comparison Method 1	94.82
Comparison Method 2	95.26
Comparison Method 3	96.04

**Table 5:** Training and test samples under depression angle variance.

	Depression angle (°)	2S1	BDRM2	ZSU23/4
Training set	17	299	298	299
Test set	30	288	287	288
	45	303	303	303

**Table 6:** Recognition results of different methods at different depression angles.

Method type	Average recognition rate (%)	
	30°	45°
Proposed	97.12	73.13
Comparison Method 1	95.82	66.24
Comparison Method 2	96.04	68.28
Comparison Method 3	96.84	70.56

## Data Availability

The dataset used to support this study is available upon request.
